# Efficacy and Safety of Endoscopic Tympanic Membrane Catheterization Plus Ofloxacin Ear Drops in the Treatment of Secretory Otitis Media in Infants and Toddlers

This article has been retracted.

**DOI:** 10.1155/2022/3732243

**Published:** 2022-07-21

**Authors:** Zhang Zhao, Zhuxiang Chen

**Affiliations:** Hubei No. 3 People's Hospital of Jianghan University, Wuhan, Hubei 430033, China

## Abstract

**Objective:**

To investigate the efficacy and safety of endoscopic tympanic membrane catheterization and ofloxacin ear drops in the treatment of secretory otitis media in infants and toddlers.

**Methods:**

A total of 80 children suffering from secretory otitis media who underwent treatment in our hospital from July 2018 to April 2020 were divided into the control group (*n* = 40) and experimental group (*n* = 40) by randomization. The control group was treated with endoscopic tympanic membrane catheterization alone, while the experimental group was treated with ofloxacin ear drops based on the same treatment as the control group. The treatment effect, air conduction hearing level, clearance rate of pathogenic bacteria secreted by the ear canal, recurrence rate, and adverse reactions were compared between the two groups.

**Results:**

The treatment in the experimental group led to a significantly better outcome than that in the control group (*P* < 0.05). After treatment, a substantially improved air conduction hearing level in the experimental group was observed (*P* < 0.001). A chi-square test showed a significantly higher clearance rate of pathogenic bacteria secreted from the ear canal of the children in the experimental group compared to that of the control group (*P* < 0.05). The treatment in the experimental group resulted in a lower recurrence rate and adverse reaction rate as compared to the control group (*P* < 0.05).

**Conclusion:**

Concurrent endoscopic tympanic membrane catheterization and ofloxacin ear drops showed excellent efficacy in the treatment of secretory otitis media in infants and toddlers. The therapy offers promising solutions for the improvement of hearing level, increase of clearance rate of pathogenic bacteria secreted from the ear canal, and decrease of disease recurrence and adverse reactions during treatment.

## 1. Introduction

Secretory otitis media is a common disease in clinical pediatrics among infants and toddlers, whereby delayed treatment causes hearing loss [1]. Secretory otitis media is mainly characterized by ear aches, tinnitus, ear discomfort, hearing loss, and middle ear effusion [2]. Due to the underdevelopment of muscles and cartilage of the eustachian tube in infants and toddlers, the muscles of the body are prone to weak contractions, leading to the pressure resulting from the collapse of the cartilage tube and inducing secretory otitis media [3]. Li et al. [4] highlighted that secretory otitis media in infants and toddlers entails adverse effects on their language competence, intelligence, and development. Based upon ventilation and drainage of effusion, current treatment regimens of secretory otitis media in infants and toddlers mainly include endoscopic tympanic membrane catheterization for the mitigation of the clinical symptoms. However, some clinical studies have concluded that endoscopic tympanic membrane catheterization is associated with a high disease recurrence rate. Some scholars believe that this may result from the lack of adequate inflammation control in children, thereby resulting in complications such as otorrhea in children [5]. Antibacterial ear drops can effectively help children with otitis media to control the body's inflammatory response. Telipid ear drops are a novel type of quinolone broad-spectrum antibacterial drug [6]. This study aims to investigate the effect of endoscopic tympanic membrane catheterization and Telipid with the hypothesis that it would showcase higher efficacy in secretory otitis media.

## 2. Materials and Methods

### 2.1. Baseline Data

A total of 80 children with secretory otitis media who were treated in our hospital from July 2018 to April 2020 were equally assigned into the control group (*n* = 40) and experimental group (*n* = 40) by randomization. In the control group, the children aged from 2 months to 3 years, and their course of disease was 5–27 days. In the experimental group; the children aged from 3 months to 3 years, and their course of the disease was 4–28 days. This study was reviewed and approved by the Medical Ethics Committee of Hubei NO.3 People's Hospital of Jianghan University, No.187971, and all the families of the children were informed about the study and gave assent.

### 2.2. Inclusion and Exclusion Criteria

Inclusion criteria: (1) patients aged less than 4 years; (2) patients met the clinical diagnostic criteria for secretory otitis media; (3) patients had no allergic reactions to the relevant drugs in this study and could undergo full treatment. Exclusion criteria: (1) patients with nasal inflammatory diseases; (2) patients who have undergone other treatment regimens; (3) Patients who could not follow the modalities of the study.

### 2.3. Methods

Both groups underwent endoscopic tympanic membrane catheterization. The specifics were as follows: the patient was placed in a supine position, the outer ear was sterilized with ethanol, and the tympanic membrane was anesthetized with tetracaine cotton pads (manufacturer: Yuekang Pharmaceutical Group Co. Ltd.); an otoscope was inserted through the external auditory canal, an arc-shaped incision was performed in the anterior and lower quadrants of the tense part of the tympanic membrane, the tympanic membrane was incised, and the effusion in the tympanic membrane was drained. A T-shaped silicone ventilation tube was subsequently placed on the curved incision for the *R* to be located on the edge of the tympanic membrane incision, and the outer ear channel was sealed with a sterile cotton ball. The catheter was kept for 3 months. The children in the experimental group were treated with ofloxacin ear drops (manufacturer: Shenzhen Wanhe Pharmaceutical Co. Ltd., approval number: H20090024, specification: 10 ml) during the intubation treatment, 3 times/d, about 10 drops/time, for a total of 3 weeks of ear drop treatment.

### 2.4. Observation Indicators

1. After 6 months of intubation, the therapeutic effect was observed. Cured: the symptoms of the child's ear discomfort disappeared, and the color of the visible light cone was mostly restored to normal levels by otoscopy; improved: the symptoms of the child's ear discomfort were relieved, and the color of the visible light cone was improved; ineffective: symptoms such as ear discomfort did not improve, or were even exacerbated. Total effective rate = (cured + improved)/total number of cases × 100%.
2. Air conduction hearing level after 6 months with intubation. The pure-tone hearing threshold was used to test the hearing levels of the children with set frequencies of 0.5, 1.0, and 2.0 kHz after treatment, and documented by the medical staff in our hospital. Average threshold levels of 0.5, 1.0, and 2.0 kHz: −10–15 dB is normal; 16–25 dB is the minor hearing loss range; 26–40 dB is the mild hearing loss range; 41–55 dB is the moderate hearing loss range; 56–70 dB is the moderate to severe hearing loss range; 71∼90 dB is the severe hearing loss range; above 91 dB is extreme hearing loss range.
3. Clearance rate of secreted pathogenic bacteria after 6 months with intubation. Tympanic membrane puncture was routinely performed to extract the effusion and placed on a glass slide, and the Wright stain was used for cytological observation. The total number of pathogenic bacteria in the two groups was recorded by the medical staff of our hospital to calculate the clearance rate of secretory pathogenic bacteria. Bacterial clearance rate = The total number of pathogenic bacteria after treatment/The total number of pathogenic bacteria before treatment × 100%.
4. The recurrence rate and the incidence of adverse reactions within 3 months after extubation. The recurrence of the disease was recorded by the medical staff in our hospital; and the possible adverse reactions sustained by the children during the treatment included infection, tube detachment, tube blockage, and otorrhea.

### 2.5. Statistical Analysis

SPSS21.0 was used for data analysis. Measurement data are expressed as (*x* ± *s*) and were analyzed by the independent samples *t*-test; enumeration data are expressed as the number of cases (rate), and were compared using the chi-square test. Statistical significance was set at *P* < 0.05.

## 3. Results

### 3.1. Patient Profile

There were 26 males and 14 females in the control group, with an average age of (1.57 ± 0.72) years and an average course of (17.32 ± 2.81) days. There were 24 males and 16 females in the experimental group, with an average age of (1.60 ± 0.69) years and an average course of (17.44 ± 2.75) days. The baseline data between the two groups of patients were comparable (*P* > 0.05), as listed in Table 1.

### 3.2. Treatment Effects

In the control group, 11 cases of children were cured, 18 cases were improved, and 11 cases were invalid; 26 cases of children in the experimental group were cured, 12 cases were improved, and 2 cases were invalid. The total treatment efficiency of children in the control group was 73% (29/40), which was lower than that of the experimental group which was 95% (38/40). The difference was deemed statistically significant (*P* < 0.05, Table 2).

### 3.3. Air Conduction Hearing Levels

After treatment, air conduction hearing levels for children in the control group of 0.5 kHz, 1.0 kHz, and 2.0 kHz are, respectively, (21.28 ± 3.27) dB, (17.35 ± 2.57) dB, and (13.21 ± 1.79) dB, all of which are higher than the data in the experimental group, (11.42 ± 1.56) dB, (13.00 ± 10.22) dB, (7.42 ± 0.86) dB. The difference was statistically significant (*P* < 0.001), as shown in Table 3.

### 3.4. Clearance Rate of Pathogenic Bacteria Secreted from the Ear Canal

The pathogen clearance rate of the children in the control group after treatment was 62% (34/55), while the clearance rate of pathogenic bacteria in the experimental group was 89% (50/56). The chi-square test showed a significantly higher clearance rate of pathogenic bacteria secreted from the ear canal of the children in the experimental group compared to the control group (*P* < 0.05), as listed in Table 4.

### 3.5. Recurrence and Adverse Reactions

In the experimental group, the recurrence rate of children was 5% (2/40) and the total incidence of adverse reactions was 5% (2/40), both lower than 20% (8/40) and 23% (9/40) of control group children. The difference was deemed statistically significant (*P* < 0.05, Table 5).

## 4. Discussion

Secretory otitis media has certain particularities in infants and toddlers. Given the incomplete development of infants and toddlers' autoimmune organs and tissues, immune function and resistance are relatively poor, which could entail upper respiratory tract infection. Coupled with the short curvature and small curvature of the Eustachian tube and the immature development of the tensor veli muscle in infants and toddlers, secretory otitis media could manifest itself easily [7]. Infants and toddlers are in a critical period of language and intellectual development. Delayed and ineffective treatment would substantially hinder the development of infants' and toddlers' vocal and intelligence functions [8]. Despite unclear pathogenesis, the contributing factor of adenoid hypertrophy has been identified. The clinical manifestations of secretory otitis media mainly include hearing loss, sleep snoring, sinusitis, and tonsil hypertrophy. In severe cases, children may suffer from permanent hearing loss, substantially compromising their physical and mental health [9]. Adenoid hypertrophy is one of the common clinical manifestations of secretory otitis media, which can entail nasopharyngeal secretion regurgitation in children, aggravating the auditory diseases and increasing the inflammatory mediators in children's body and cell number. Moreover, it raises the risk of local inflammation in children [10]. The clinical treatment for secretory otitis media includes two surgical and nonsurgical treatment options. Among them, nonsurgical treatments include nasal antiallergy, eustachian tube inflating, middle ear antibacterial, and anti-inflammatory; however, these methods could easily result in recurrence or secondary conditions [11]. Surgical treatment mainly includes myringotomy, myringotomy, and myringocentesis. With comprehensive clinical research and application of otoscope technology, the technology of tympanostomy tube placement under otoscope has gained maturity, and its operation can effectively obviate the risk of the tympanic membrane and external auditory canal damage caused by conventional tympanostomy tubes placement. The method can reasonably select and control the incision method and size of children [12]. On the one hand, through ear endoscopy, medical practitioners are capable of comprehending the degree and characteristics of the effusion in the tympanic cavity of children [13]. On the other hand, endoscopic otoscope surgery can yield a clearer operative field through the imaging system, which enables the tympanic membrane cannulation to be performed visually, thereby shortening operating time, and reducing the number of operative steps. The injury to the children's ears reduces their postoperative pain, thereby significantly improving treatment safety [14]. However, some clinical studies found that the disease recurrence rate of children with secretory otitis media treated only by endoscopic tympanic membrane catheterization is still high [15].

Antibacterial ear drops can effectively help children with otitis media in controlling the body's inflammatory response. Telipidal ear drops are a new type of quinolone broad-spectrum antibacterial drug, which has been clinically proved to exert significant therapeutic effects on various infectious diseases. Novotny et al. [16] pointed out that Telipidal ear drops have high antibacterial activity and good stability, and its application in combination with tympanostomy tube placement under ear endoscopy can relieve the secretion of children suffering from secretory otitis media. The pathogenic bacteria have an efficient inhibitory effect, thereby blocking the infectious source in children and markedly reducing the disease recurrence rate and the incidence of related adverse reactions in children [17]. The new type of quinolone broad-spectrum antibacterial drugs can reduce the drug tolerance of bacteria, greatly improve the bactericidal activity of drugs, and effectively curb the generation of drug resistance. It acts on bacterial type II-A topoisomerases (DNA rotase and topoisomerase IV) [2–4]. Studies have shown that the process of bacterial DNA replication is essential for the growth and survival of bacteria, and this process requires the combined action of DNA rotase and topoisomerase IV [4]. The treatment of new quinolones with broad-spectrum antibacterial drugs forms a “drug-topoisomerase-DNA” triple complex interaction and promotes the molecular processing law of the complex to release broken DNA, thereby deepening the understanding of the bactericidal mechanism of quinolones. Based on this theory, a high-throughput screening system for small-molecule bactericidal synergists and dormant bacteria efficiently killing quinolone molecules is initially established to reduce clinical drug resistance and promote the development of new drugs. We compared the therapeutic effect, air conduction hearing level, clearance rate of pathogenic bacteria secreted from the ear canal, recurrence and adverse reactions between the two groups of children. The results showed that the therapeutic effect of the children in the experimental group outperformed the results shown by the children in the control group. After treatment, the air conduction hearing level of the children in the experimental group was markedly better than that of the children in the observation group; the clearance rate of pathogenic bacteria secreted from the ear canal of the children in the experimental group was significantly better than that of the children in the control group; the disease recurrence rate of the children in the experimental group and the incidence of adverse reactions was significantly lower than that of the control group. The results of this study were consistent with those of the previous study [18]. This finding may be due to the fact that with the tympanostomy tubes placement under otoscope, it is impossible to completely circumvent the infection caused by the sewage entering the tympanic cavity and ear canal even excluding the substandard disinfection steps by doctors during the operation and the retrograde pathogenic bacteria infection or secondary eustachian tube caused by the operation [19]. Therefore, the use of Telipidal ear drops is necessary for adjuvant treatment, which can produce a good secretion of pathogenic bacteria in children. Only by suppressing the pathogenic bacteria in children can we truly and effectively remove the infection lesions, which is an important step in reducing the disease recurrence rate and the incidence of adverse reactions in children [20].

With the progress in research, although Western medicine treatment has curative effects, it is mostly treated with antibiotics, intratympanic injections, nasal drops, etc., However, these treatments are not ideal, and long-term use of antibiotics and glucocorticoids can cause certain adverse reactions; tympanic tube placement can result in chronic purulent otitis media, secondary cholesteatoma, permanent perforation of the tympanic membrane, tympanic hardening, and other complications, and cannot fundamentally solve the issue of poor eustachian tube function. Recently, a patent shows that traditional Chinese medicine treats chronic secretory otitis media, liver, yin, kidney, and yin deficiency in children. Traditional Chinese medicine includes Baishihua, Penzi grass, long-petal borage moss, inverted umbrella, single grass, Yunnan Cheqian, Huajian grass, cordierleaf mountain plum blossom, ice grass root, long-leaf purple beads, grass cistanche, great soul grass, ghost feather arrow, white wood, slap grass, grass vine, walking thousands of miles alone, and ancient hook vine. The combination of traditional Chinese medicine and Western medicine treatment methods can overcome the side effects caused by Western medicine, improve the efficacy, shorten the treatment time, and have a good effect on chronic secretory otitis media in children with liver and kidney yin deficiency. However, this applies to children who can take it on their own. It is not suitable for infants and toddlers included in this study, and the treatment methods of this study are still necessary.

## 5. Conclusion

Endoscopic tympanic membrane catheterization plus Telipid is effective in the treatment of secretory otitis media in infants and toddlers. The therapy offers promising solutions for the improvement of hearing levels, an increase in clearance rates of pathogenic bacteria secreted from the ear canal, and a decrease in recurrence of disease and adverse reactions during treatment. Therefore, it warrants clinical application. Future research will consider more comprehensive factors, including the use of nonstatistical antibiotics for infants and toddlers of different ages, as well as multicenter research.

## Figures and Tables

**Table 1:** Comparison of general data.

Index	Control group (*n* = 40)	Experimental group (*n* = 40)	*t*/*x*^2^	*P* value
Gender				
Male	26	24	0.213	0.644
Female	14	16		
Age (year, *x* ± *s*)	1.57 ± 0.72	1.60 ± 0.69	0.190	0.850
Course of disease (month, *x* ± *s*)	17.32 ± 2.81	17.44 ± 2.75	0.193	0.847

**Table 2:** Comparison of treatment effects.

	Control group (*n* = 40)	Experimental group (*n* = 40)	*X* ^2^	*P* value
Cured	11	26		
Improved	18	12		
Ineffective	11	2		
Total effectiveness (%)	29 (73)	38 (95)	7.440	0.006

**Table 3:** Comparison of air conduction hearing levels ($\bar{X}\pm s$, dB).

Groups	0.5 kHz	1.0 kHz	2.0 kHz
Control group (*n* = 40)	21.28 ± 3.27	17.35 ± 2.57	13.21 ± 1.79
Experimental group (*n* = 40)	11.42 ± 1.56	10.22 ± 1.13	7.42 ± 0.86
*t*	17.212	16.062	18.44
*P* value	<0.001	<0.001	<0.001

**Table 4:** Comparison of clearance rates of pathogenic bacteria secreted from the ear canal.

	Control group (*n* = 40)	Experimental group (*n* = 40)	X^2^	*P* value
The total number of pathogenic bacteria before treatment	55	56		
The total number of pathogenic bacteria after treatment	34	50		
Clearance rate (%)	62	89	19.705	<0.001

**Table 5:** Comparison of recurrence and adverse reactions.

	Control group (*n* = 40)	Experimental group (*n* = 40)	*X* ^2^	*P* value
Recurrence rate (%)	8(20)	2(5)	4.114	0.043

Adverse reaction				
Infection	4	1		
Tube detachment	2	1		
Tube plugging	2	0		
Otorrhea	1	0		
Total incidence (%)	9 (23)	2 (5)	5.165	0.023

## Data Availability

No data were used to support this study.

## References

[1] Hoberman A., Preciado D., Paradise J. L. (2021). Tympanostomy tubes or medical management for recurrent acute otitis media. *New England Journal of Medicine*.

[2] Satoh C., Toizumi M., Nguyen H. A. T. (2021). Prevalence and characteristics of children with otitis media with effusion in Vietnam. *Vaccine*.

[3] Luu K., Park J., Shaffer A. D., Chi D. H. (2020). Long-term otitis media outcomes in infants with early tympanostomy tubes. *Otolaryngology—Head and Neck Surgery*.

[4] Li L., Mao Y., Hu N. (2021). The effect of balloon dilatation eustachian tuboplasty combined with grommet insertion on the structure and function of the eustachian tube in patients with refractory otitis media with effusion. *Annals of Palliative Medicine*.

[5] Takai S., Nomura K., Oda K. (2021). Clinical factors associated with the outcomes of long-term middle ear ventilation tube insertion in pediatric patients. *Ear, Nose, & Throat Journal*.

[6] Liu J., Wang X. (2021). Ofloxacin-loaded niosome-laden contact lens: improved properties of biomaterial for ocular drug delivery. *AAPS PharmSciTech*.

[7] Skovbjerg S., Roos K., Andersson M. (2020). Inflammatory mediator profiles in secretory otitis media in relationship to viable bacterial pathogens and bacterial and viral nucleic acids. *Journal of Interferon and Cytokine Research*.

[8] Tengroth B., Lohmander A., Hederstierna C. (2020). Hearing thresholds in young children with otitis media with effusion with and without cleft palate. *The Cleft Palate-Craniofacial Journal*.

[9] Xu Z., Han C., Dang Z., Huang T., Li Z., Huang Y. (2021). The bacteriological characteristics and drug resistance of the nasopharyngeal region in 311 cases of adenoid hypertrophy with secretory otitis media. *Lin Chung Er Bi Yan Hou Tou Jing Wai Ke Za Zhi*.

[10] Sogebi O. A., Oyewole E. A., Ogunbanwo O. (2021). Asymptomatic otitis media with effusion in children with adenoid enlargement. *Journal of the National Medical Association*.

[11] Aluko A. A. (2019). Use of phenol as a local anaesthetic for adult grommet insertion in resource-limited settings: a preliminary report. *International Journal of Otolaryngology*.

[12] Lei L., Wang D., Hao X. (2020). Therapeutic outcome and complication management of grommet insertion for radiotherapy induced otitis media with effusion. *Lin Chung Er Bi Yan Hou Tou Jing Wai Ke Za Zhi*.

[13] Mohammed H., Qureshi M. H., Yates P. (2021). Outcomes of examination under anaesthesia of post-nasal space and grommet insertion in adults presenting with otitis media with effusion. *Journal of Laryngology and Otology*.

[14] Kaya S., Keseroglu K., Tokgoz S. A., Barmak E., Saylam G., Korkmaz M. H. (2021). Multifrequency multicomponent tympanometry in children with a history of ventilation tube insertion. *International Journal of Pediatric Otorhinolaryngology*.

[15] Skarzynska M. B., Gos E., Czajka N., Sanfis M. D., Skarzynski P. H. (2021). Effectiveness of surgical approach of insertion ventilation tubes (tympanostomy) and adenoidectomy in Comparison with non-surgical approach (watchful waiting approach) in children at the age between 1 and 6 and who suffer from otitis media with effusion (OME) in 12-month period of observation-the retrospective analysis. *International Journal of Environmental Research and Public Health*.

[16] Novotny L. A., Chiang T., Goodman S. D., Elmaraghy C. A., Bakaletz L. O. (2021). Humanized anti-DNABII fab fragments plus ofloxacin eradicated biofilms in experimental otitis media. *The Laryngoscope*.

[17] Kaur G., Singh N., Rajor A. (2021). Ofloxacin adsorptive interaction with rice husk ash: parametric and exhausted adsorbent disposability study. *Journal of Contaminant Hydrology*.

[18] Huang Y. M., Li G., Li M. (2021). Kelp-derived N-doped biochar activated peroxymonosulfate for ofloxacin degradation. *Science of the Total Environment*.

[19] Chen H., Wang J. (2021). Degradation and mineralization of ofloxacin by ozonation and peroxone (O_3_/H_2_O_2_) process. *Chemosphere*.

[20] Alshahni M. M., Alshahni R. Z., Fujisaki R. (2021). A case of topical ofloxacin-induced otomycosis and literature review. *Mycopathologia*.

